# Meta-analysis of contrast-enhanced ultrasound and contrast-enhanced harmonic endoscopic ultrasound for the diagnosis of gallbladder malignancy

**DOI:** 10.1186/s12911-020-01252-5

**Published:** 2020-09-17

**Authors:** Xue Liang, Xiang Jing

**Affiliations:** Department of Ultrasound, Tianjin Third Central Hospital, Tianjin Institute of Hepatobiliary Disease, Tianjin Key Laboratory of Artificial Cell, Artificial Cell Engineering Technology Research Center of Public Health Ministry, No. 83, Jintang Road, Hedong District, Tianjin, 300170 China

**Keywords:** Gallbladder, Contrast-enhanced ultrasound, Endoscopic ultrasonography, Malignant lesions, Diagnosis, Meta-analysis

## Abstract

**Background:**

The diagnosis between benign and malignant gallbladder lesions is sometimes difficult. The objective of this study is to assess whether contrast-enhanced ultrasound (CEUS) and contrast-enhanced harmonic endoscopic ultrasound (CH-EUS) can be an accurate method for detecting gallbladder malignancy and to determine which imaging signs can be indicative of malignancy.

**Methods:**

A study search of PubMed, Elsevier, and Sciencedirect was performed in May 2019. The pooled sensitivity, specificity, diagnostic odds ratio (DOR), and summary receiver operating characteristic (SROC) curve were used to examine the accuracy of CEUS and CH-EUS.

**Results:**

Twenty-one studies were included in the meta-analysis. The pooled sensitivities of CEUS and CH-EUS were 0.81 (0.75–0.86) and 0.92 (0.86–0.95); the specificities were 0.94 (0.90–0.96) and 0.89 (0.69–0. 97); the DORs were 64 (32–127) and 89 (22–354); and the area under the SROC curves were 0.90 (0.87–0.92) and 0.92 (0.90–0.94). On CEUS, the diagnostic criterion for gallbladder malignancy according to four features were analyzed. Sensitivity and specificity were 0.75 (0.65–0.83) and 0.98 (0.85–1.00) for integrity of gallbladder wall; 0.69 (0.55–0.81) and 0.89 (0.77–0.95) for heterogeneous enhancement; 0.81 (0.71–0.88) and 0.88 (0.76–0.94) for irregular vessels; and 0.81 (0.66–0.91) and 0.75 (0.59–0.86) for washout time within 28 s. On CH-EUS, heterogeneous enhancement could be indicative of malignant lesions with a sensitivity of 0.94 (0.85–0.97); and the specificity was 0.92 (0.71–0.98).

**Conclusions:**

CEUS and CH-EUS are promising and reliable imaging modalities with a high sensitivity and specificity for the diagnosis of gallbladder malignancy. CH-EUS might be more sensitive than CEUS with a higher sensitivity. In addition, irregular tralesional vessels and washout time within 28 s on CEUS and heterogeneous enhancement on CH-EUS are indicative of malignancy. However, larger scale and well-designed studies are warranted to verify our results.

## Background

Conventional ultrasound (US) is the first-line imaging method for diagnosis of gallbladder (GB) diseases because of its advantages over other imaging modalities such as computed tomography or magnetic resonance imaging, including real-time scanning, easy manipulation, cost-effectiveness, no ionizing radiation, high resolution, and repeatability [1, 2]. However, the diagnosis between benign and malignant GB lesions by using US is often challenging. Many GB carcinomas are not diagnosed preoperatively because of nonspecific symptoms or asymptomatic presentation unless the cancer invades adjacent organs, especially the early GB carcinomas. In patients with early GB cancer, thickening of the wall may be the only detectable imaging sign; and US usually makes a poor diagnosis because wall thickening can also occur in many benign lesions, such as adenomyomatosis [3, 4]. In addition, the accuracy of conventional US might be limited with the inappropriate position of the artifacts of imaging and insufficiency for obtaining low speed blood flow information in the GB lesions. In order to improve diagnostic accuracy and reduce unnecessary surgery, it’s important to develop new US modalities to precisely differentiate malignant from benign lesions.

In recent years, contrast-enhanced ultrasound (CEUS) has been used for the diagnosis of GB diseases and is considered as a valuable complement to conventional US. The use of contrast agents allows the depiction of small vessels and improves the characterization of the microvasculature inside the organ [5]. .It is well accepted that lesions larger than 10 mm are indicative of malignancy, and cholecystectomy is needed [6]. However, Liu et al. and Xu et al. have reported that lesions less than 10 mm are also seen in some malignancy [7, 8]. Actually, except for lesion size, other characteristics such as vascularity, enhancement pattern, and washout time may be helpful for differentiation due to the depiction of macro- and micro- circulation in CEUS, and thereby increasing the diagnostic accuracy.

Contrast-enhanced harmonic endoscopic ultrasound (CH-EUS) is another novel technology that assesses both the microvasculature and parenchymal perfusion by selectively depicting the signals derived from the US contrast agent [5]. Endoscopic ultrasonography is considered to be superior to US for depiction of GB lesions and provides high-resolution images [9]. Under some circumstances, distinguishing organs on percutaneous abdominal US can be difficult, particularly if a patient has a large amount of subcutaneous fat or intestinal gas. Endoscopic ultrasonography from the lumen of the stomach or duodenum can be used to visualize organs more clearly due to proximity of the ultrasound probe to the region of interest and its high spatial resolution [10, 11]. Therefore, the application of contrast agents in endoscopic ultrasonography should be a powerful diagnostic approach.

However, diagnostic evidence of CEUS and CH-EUS for distinguishing GB carcinomas is still limited, and additional information about the two novel methods is required. In the present study, we assessed whether CEUS and CH-EUS could be an accurate method for detecting GB malignant lesions. We also determined which imaging signs could be indicative of malignancy based on assessment of the vessel and the perfusion features.

## Methods

This meta-analysis was conducted according to the guidelines of the Preferred Reporting Items for Systematic Reviews and Meta-analysis statement.

### Search strategy

Literature search was performed in the PubMed, Embase, Elsevier, and Siencedirect to identify all the relevant studies published before May 2019. The keywords were used for identification as the following: gallbladder, contrast-enhanced, ultrasound, malignant lesions, carcinoma, as well as their abbreviations and synonyms and combined search terms. In addition, references of the included studies were also checked to cover more eligible papers. Potentially relevant articles were firstly evaluated by reviewing the titles and abstracts, and then each full text was read to further identify the included studies.

### Inclusion and exclusion criteria

The selected publications must meet all criteria as the following: (1) use of CEUS or CH-EUS in the diagnosis of malignant GB lesions; (2) comparison of the diagnostic results of the tested imaging techniques with a reference standard; (3) sufficient data to construct a 2 × 2 contingency table for calculation; and (4) articles written in English. Review studies, case reports, comments, editorial articles were excluded. Studies published in abstract form only were also excluded. If more than one report were same in the patients groups, the article with the most sufficient data was included. Studies eliminating samples with missing values were acceptable when large datasets are available and missing values occur only in a small percentage of samples [12, 13].

### Data extraction

Data from each included studies were reviewed and abstracted into an Excel spreadsheet by two authors independently. The data form was predefined and standardized, and the extracted information included first author, publication year, country, study design, sample size, patients baseline characteristic (age, gender, type of disease), gold reference standards, contrast agents, mechanical index (MI), and imaging interpretation method (blinded or unblinded). In each study, data regarding diagnostic accuracy of imaging modalities were also abstracted, and values for true-positive (TP), true-negative (TN), false-positive (FP), and false-negative (FN) were directly recorded or calculated, and 2 × 2 contingency tables were conducted. Differences between reviewers were resolved by discussion until agreement was reached.

### Quality assessment

The methodological quality of each included studies was assessed by the same two authors independently, in accordance with the Quality Assessment of Diagnostic Accuracy Studies (QUADAS-2) [14]. The QUADAS-2 tool consists of four domains: patient selection, index test, reference standard, and flow and timing. For each item, the risk of bias was ranked as “low” if reported; “high” if not reported; “unclear” if no adequate information was provided. Disagreements were also resolved by discussion.

### Statistical analysis

All the statistical analysis was conducted using Stata, version 15.0 (Stata Corporation, College Station, TX) and Review Manage 5.3 software (The Nordic Cochrane Centre, The Cochrane Collaboration). The pooled data of sensitivity, specificity, and DOR with their 95% CIs, were calculated to determine the diagnostic performance of CEUS and CH-EUS in the detection of GB carcinoma. SROC were constructed to evaluate the effect of sensitivity and specificity. The AUC of SROC was used to analyze the diagnostic accuracy of determined groups, and a higher AUC value reveals a better test result.

The heterogeneity of the individual studies was estimated by the Q statistic of the Chi-square values test and the inconsistency index (I^2^). A significant heterogeneity was present if I^2^ ≥ 50%, and random effect was chosen to pool the data; otherwise, a fixed-effect model was used. For evaluation of diagnostic studies, one of the most potential sources of heterogeneity is the threshold effect, which was caused by the different cut-offs or thresholds to define a positive or negative test result. Spearman correlation coefficients between the logit of sensitivity and the logit of (1-specificity) were calculated to assess the threshold effect. A strong positive correlation was indicative of a threshold effect, *P* < 0.05. In addition, a meta-regression analysis and a subgroup analysis were performed to disclose other variance that could result in heterogeneity among studies and factors that affect the overall diagnostic accuracy, which can mathematically represent the interaction between different variables as a statistical method [15, 16].

Continuous variable in this meta-analysis, like time, was estimated by weighted mean differences (WMD) and its 95% CI. Publications bias was assessed by the Deeks funnel plot and an asymmetry test, and *P* value greater than 0.05 was considered no significant publication bias.

## Results

### Study identification

A total of 2063 potentially relevant articles were identified in the initial search stage. Most of these papers were excluded due to titles and abstracts. Only 159 studies were chosen for full-text review. Further identification excluded 94 articles that were not of interest for this meta-analysis and 44 papers that failed to provide sufficient or related data for the calculation of diagnostic accuracy. Finally, 21 articles satisfying the inclusion criteria were included and analyzed [2, 7, 8, 17–34]. The demonstration of study search flow can be seen in Fig. 1.

**Fig. 1:** Flowchart of study selection

### Study characteristics

The study characteristics of all included studies were demonstrated in Table 1. Among these 21 selected studies, 15 studies evaluated the diagnostic role of CEUS, and 6 studies explored the diagnostic performance of CH-EUS. A total of 1695 patients were analyzed. The groups of CEUS and CH-EUS included 1237 and 458 patients, respectively. All studies applied the method of blinded interpretation of tested imaging modality, except three trails that did not mention the assessment methods. Detailed information regarding sample size, age, gender, reference standard, contrast medium and MI in individual study are shown in Table 1.

**Table 1:** Characteristics of the included studies

Author	Year	Region	Study design	Patients	Age	Male/Female	Standard reference	Contrast Agent	MI	Imaging modality
Chen	2017	China	Retrospective	72	64 ± 11	22/11	Pathological results	SonoVue	< 0.1	CEUS
Choi	2013	Korea	Retrospective	90	52.7 (35–83)	NA	Pathological results	SonoVue	NA	CH-EUS
Hirooka	1998	Japan	Retrospective	38	NA	NA	Histological results	Albunex	NA	CH-EUS
Imazu	2014	Japan	Retrospective	36	63.9 ± 10.3	NA	Histological results	Sonazoid	0.25–0.3	CH-EUS
Inoue	2007	Japan	Retrospective	90	67 (51–84)	55/35	Histological results	Levovist	NA	CEUS
Kamata	2017	Japan	Retrospective	125	61 (19–82)	67/58	Histological results	Sonazoid	0.3	CH-EUS
Leem	2018	Korea	Retrospective	145	55.4 ± 15.2	58/87	Histological results	SonoVue	0.2	CH-EUS
Liu	2012	China	Prospective	192	52 (15)	83/109	Pathological results	SonoVue	0.05–0.20	CEUS
Liu	2015	China	Prospective	83	50.29 ± 13.16	37/46	Histological results	SonoVue	0.06	CEUS
Miwa	2018	Japan	Retrospective	36	65.7 ± 12.6	17/19	Pathological results	Sonazoid	0.8–1.2	CEUS
Numata	2007	Japan	Retrospective	33	62 (26–87)	20/13	Histological results	Levovist	1.0–1.6	CEUS
Serra	2018	Italy	Retrospective	39	NA	NA	Pathological results	SonoVue	NA	CEUS
Sugimoto	2016	Japan	Retrospective	24	61.8 ± 15.1	8/16	Pathological results	Sonazoid	NA	CH-EUS
Sun	2015	China	Retrospective	34	54.7 ± 18.8	16/18	Histopathological results	SonoVue	< 0.2	CEUS
Xie	2010	China	Retrospective	80	54.6 ± 13.1	37/43	Pathological results	SonoVue	0.08–0.10	CEUS
Xu	2014	China	Prospective	159	55.6 ± 14.1	76/83	Histopathological results	SonoVue	< 0.2	CEUS
Yuan	2015	China	Retrospective	37	NA	NA	Pathological results	SonoVue	0.05–0.10	CEUS
Yuan	2018	China	Retrospective	75	56.6 ± 10.5	34/41	Histopathological results	SonoVue	0.05–0.10	CEUS
Zhang	2018	China	Retrospective	103	42.5 ± 10.6	47/56	Pathological results	SonoVue	NA	CEUS
Zheng	2013	China	Prospective	116	49.6 ± 14.5	47/69	Pathological results	SonoVue	0.05–0.20	CEUS
Zhuang	2017	China	Retrospective	88	48.8 ± 14.5	41/47	Pathological results	SonoVue	0.08–0.10	CEUS

*NA* not applicable; *MI* Mechanical index; *CEUS* contrast-enhanced ultrasound; *CH-EUS* contrast-enhanced endoscopic ultrasonography

### Quality assessment

Figure 2 presents the results of the quality assessment of all included studies according to QUADAS-2. No high risk of bias was found in four items. Unclear risk of bias in the item of “patients selection” was observed because inappropriate exclusions was unclear in many studies. In the “index test” category, a pre-specified threshold was not mentioned in a part of study that caused the unclear risk of bias. For the item of “reference standard”, only a minority of trials failed to introduce the blinded interpretation. All analyzed studies presented low risk of bias concerning “flow and timing” category.

**Fig. 2:** Quality assessment of the included studies

### Diagnostic accuracy of CEUS

In terms of the diagnostic quality of CEUS in differentiating malignant and benign GB diseases, the pooled sensitivity was 0.81 (95% CI: 0.75–0.86) and the pooled specificity was 0.94 (95% CI: 0.90–0.96) (Fig. 3a). The DOR was 64 (95% CI: 32–127). The AUC of SROC was 0.90 (95% CI: 0.87–0.92) (Fig. 3b), indicating its good ability to diagnose malignant GB lesions. Further analysis of Spearman correlation coefficients revealed that no threshold effect was present among these studies (*P* = 0.60). Concerning a relatively slight heterogeneity was found in sensitivity (I^2^ = 38.28%) and a significant inconsistency in specificity (I^2^ = 67.30%), subgroup analysis according to inclusion criteria about lesion diameter and duration of imaging were conducted and revealed high sensitivity and specificity with lower I^2^ values, particularly in the subgroups of time ≥ 3 min and lesions ≥10 mm. The results of these subgroups were shown in Table 2.

**Fig. 3:** The pooled sensitivity and specificity (**a**) and summary receiver operating characteristic curve (**b**) on CEUS for the diagnosis of gallbladder malignancy

**Table 2:** Results of meta-regression and subgroup analysis on CEUS

Subgroups	Studies	Sensitivity	I^2^ value	P value	Specificity	I^2^ value	*P* value
Imaging duration				0.08			< 0.001
< 3 min	7	0.78 (0.71–0.84)	0.00%		0.95 (0.92–0.97)	44.51%	
≥ 3 min	6	0.88 (0.73–0.95)	51.06%		0.89 (0.83–0.93)	37.25%	
Lesion size				< 0.001			0.17
< 10 mm	8	0.79 (0.71–0.85)	33.36%		0.94 (0.89–0.97)	70.22%	
≥ 10 mm	6	0.85 (0.71–0.93)	25.91%		0.91 (0.79–0.96)	56.91%	

### Discontinuity of GB wall on CEUS

Eight studies mentioned the integrity of GB wall as a diagnostic characteristic for malignant lesions on CEUS. The summary of these studies generated a sensitivity of 0.75 (95% CI: 0.65–0.83, I^2^ = 62.26%), a specificity of 0.98 (95% CI: 0.85–1.00, I^2^ = 77.73%), and a DOR of 130 (95% CI: 21–793) (Fig. 4). This sign showed the highest specificity among CEUS features. However, we could not make a successful diagnosis of malignancy independently through the observation of incomplete GB wall, though the predictor of GB wall could identify the benign lesions.

**Fig. 4:** The pooled sensitivity and specificity for the integrity of gallbladder wall on CEUS for the diagnosis of gallbladder malignancy

### Enhancement pattern on CEUS

The CEUS feature of enhancement pattern in the arterial phase on GB lesions was observed in 10 trials. The pooled sensitivity was 0.69 (95% CI: 0.55–0.81, I^2^ = 77.46%); the pooled specificity was 0.89 (95% CI: 0.77–0.95, I^2^ = 93.12%) (Fig. 5); the pooled DOR was 18 (95% CI: 7–47). Heterogeneous enhancement was frequently encountered in GB carcinoma, but homogeneous enhancement could also been seen in malignancy; and thus this perfusion imaging on CEUS only provided a limited value to the differential diagnosis.

**Fig. 5:** The pooled sensitivity and specificity for the enhancement pattern on CEUS for the diagnosis of gallbladder malignancy

### Tralesional vascularity on CEUS

When we grouped characteristics by irregular vessels among 9 studies, we found the present of vascularity allowed a good diagnostic performance on identifying malignant GB lesions with the pooled sensitivity, specificity, and DOR of 0.81(95% CI: 0.71–0.88, I^2^ = 69.26%), 0.88(95% CI: 0.76–0.94, I^2^ = 90.61%), and 30(95% CI: 17–53), respectively (Fig. 6). Most GB malignancy appeared tortuous or branched-like vascular distribution, while the vessels of GB benign lesions might show a more regular vessels in a linear or dotted shape.

**Fig. 6:** The pooled sensitivity and specificity for the tralesional vascularity on CEUS for the diagnosis of gallbladder malignancy

### Enhancement time on CEUS

There were 10 studies that reported the enhancement process using CEUS for at least 120 s. The whole enhancement change process was divided into three groups. In the group of contrast arrival time, the combination of 8 reports generated a WMD of 0.83 (95% CI: − 0.42 - 2.08, I^2^ = 75.7%) (Fig. 7a). GB malignant lesions had a tendency of “fast-in” appearance during enhancement, but no significant difference was present compared with benign group (*P* = 0.19). For the group of time to peak enhancement, the result confirmed that malignant and benign lesions reached the highest enhancement in similar time (WMD: 1.19, 95% CI: − 1.69- 4.07, I^2^ = 87.1%, *P* = 0.417) (Fig. 7b). With regard to the group of washout time, we found a significantly shorter time to hypo-enhancement on GB malignant lesions (WMD: -18.59, 95% CI: − 25.15- -12.03, I^2^ = 67.5%, *P* < 0.001) (Fig. 7c).

**Fig. 7:** The pooled weighted mean differences for the contrast arrival time (**a**), time to peak enhancement (**b**), and washout time (**c**) comparing malignant and benign lesions

Concerning that faster washout time could be an indicator for GB carcinoma detection, analysis of diagnosis accuracy was conducted according to washout time. Using a washout cut-off of 28 s, the combined CEUS sensitivity, specificity, and DOR were 0.81 (95% CI: 0.66–0.91, I^2^ = 71.11%), 0.75(95% CI: 0.59–0.86, I^2^ = 90.98%), and 13 (95% CI: 4–13), respectively (Fig. 8). These data suggested that CEUS might have a moderate diagnostic performance to detect GB carcinoma when the contrast agent washed out within 28 s.

**Fig. 8:** The pooled sensitivity and specificity for the washout time within 28s on CEUS for the diagnosis of gallbladder malignancy

### Diagnostic accuracy of CH-EUS

The application of CH-EUS in discriminating between malignant and benign GB lesions presented a pooled sensitivity of 0.92 (95% CI: 0.86–0.95, I^2^ = 57.52%) and a pooled specificity of 0.89 (95% CI: 0.69–0.97, I^2^ = 95.63%) (Fig. 9a). The DOR was 89 (95% CI: 22–354). The AUC was 0.92 (95% CI: 0.90–0.94) (Fig. 9b), indicating CH-EUS could yield an excellent value on the diagnosis of malignant GB lesions. No threshold effect was detected (*p* = 1.00). Because of small study sample size and insufficient data, we failed to conduct a subgroup analysis to further investigate the heterogeneity in sensitivity and specificity.

**Fig. 9:** The pooled sensitivity and specificity (**a**) and summary receiver operating characteristic curve (**b**) on CH-EUS for the diagnosis of gallbladder malignancy

### Enhancement patterns on CH-EUS

After pooling 4 studies that evaluated the CH-EUS feature of inhomogeneous enhancement for the GB carcinoma detection, we found CH-EUS remained highly sensitive to GB carcinoma as assessed by the pooled sensitivity of 0.94 (95% CI: 0.85–0.97, I^2^ = 61.49%), and its specificity was also high with 0.92 (95% CI: 0.71–0.98, I^2^ = 97.81%) (Fig. 10), when depending on patterns of enhancement. The DOR was 165 (95% CI: 41–663).

**Fig. 10:** The pooled sensitivity and specificity for the enhancement pattern on CH-EUS for the diagnosis of gallbladder malignancy

### Publication bias

The results of the Deeks funnel plot asymmetry test confirmed that no publication bias was observed among the studies in CEUS (*P* = 0.15), or CH-EUS (*P* = 0.62).

## Discussion

Until now, conventional US is considered the preferred method for diagnosis of GB diseases among multiple imaging modalities, not only because it is well accessible and without radiation, but also because of its good sensitivity and specificity [35]. Another method, Endoscopic ultrasonography, is considered to be superior to US for depiction of GB and provides high-resolution images which will be recommended in some special cases to improve patients management, though its characteristics of invasiveness might decrease its clinical use [9]. Sonographic differentiation among GB lesions using these imaging modalities depends largely on lesion size. However, about 60% benign lesions of GB were reported to be greater than 10 mm in some studies and caused unnecessary cholecystectomy. Meanwhile, some malignant lesions less than 10 mm increased the difficulty of diagnosis of US [7, 24, 25]. To our knowledge, the use of contrast agents can improve the diagnosis precision because of visualization of the feeding vessels to lesions and perfusion of blood, which overcomes the weakness of conventional ultrasound techniques that cannot depict tiny blood vessels and low-velocity flows [5].

Our meta-analysis which included 21 studies aimed to assess the diagnostic roles of CEUS and CH-EUS in differentiating between benign and malignant GB lesions. Except for lesion size, other features could be noticed on the screen and considered helpful for diagnosis, including the intactness of GB wall, enhancement pattern, contrast time, and intralesional vessels. Thus, we grouped by these characteristics to further investigate the two modalities.

In our study, we found that the pooled sensitivity and specificity of CEUS for GB carcinoma detection were 0.81 and 0.94, respectively, which were higher than conventional US (0.73 and 0.72, respectively) [36]. The AUC of SROC was 0.92. These data showed that CEUS could be a promising imaging modality in discriminating malignant GB lesions from benign ones, and could be widely used in clinical practice to greatly decrease unnecessary resection of GB. In the analysis of CEUS group, we noticed a notable heterogeneity in specificity (I^2^ = 67.30%). Through the results of subgroup analysis, we found that imaging duration and inclusion criteria for lesion diameter had an obvious influence on inconsistency among studies and overall diagnostic effect of CEUS. Imaging time ≥ 3 min could bring a higher sensitivity when compared with time < 3 min (0.88 vs. 0.78). It’s also estimated that longer observation could improve the overall specificity of CEUS by meta regression (*P* < 0.001). The report of Liu et al. found that the longest enhancement phase on some lesions was 150 s from contrast arrival to washout [24]. Therefore, a long enough scanning time is likely suggested to obtain more diagnostic evidence. Tumor size is another major factor affecting the diagnosis. As expected, the sensitivity decreased when lesions < 10 mm were included, which was not of interest for the early diagnosis of malignancy. It’s possible that, the presentation of malignant lesions is similar to that of benign lesions in classification system on CEUS when the lesions are small [21]; as a result, more GB carcinoma would be classified as the benign one if patients with small lesions were included, and the final diagnosis should be with cautions in this subpopulation.

Compared with conventional US, the image of CH-EUS could demonstrate the extent and depth of carcinoma invasion much better [18, 28]. Previous studies confirmed that CH-EUS is a useful method for the diagnosis of digestive diseases, but its role in the diagnosis of GB lesions is still not established [37]. According to the result of our meta-analysis, we considered CH-EUS as a promising technique in the detection of GB malignancy, with a higher sensitivity than CEUS (0.92 vs. 0.81). And its specificity and AUC were comparable with CEUS. These data indicated that CH-EUS was a sensitive modality for diagnosis of GB carcinoma.

Many experts thought that discontinuity of GB wall was an independent predictor of malignancy [2, 30]. However, during our search, the disruption of GB wall did not suggest a successful diagnosis of malignancy as expected, with a sensitivity of 0.75, but with the highest specificity of 0.98. These data mean that CEUS might accurately identify patients with benign lesions but would misclassify malignancy as benign. It has been reported that approximately 20% of GB carcinomas may not destroy the GB wall, which makes the differential diagnosis challenging and critical [38]. And GB wall discontinuity was also seen in some benign cases such as serious chronic cholecystitis. In the study of Yuan et al., the combination of incomplete of GB wall and time to hypo enhancement < 150 s presented a high sensitivity (0.93) and showed a reliable ability to detect GB malignant lesions [30]. Therefore, if the intactness of GB wall was observed in lesions, another CEUS feature should be considered to make a more accurate diagnosis.

The use of contrast agents enables the dynamic assessment and quantification of microvascularization up to capillary perfusion. CEUS are mainly applied in detection and characterization of lesions, especially benign and malignant lesions, based on differences between lesion and organ perfusion [39]. GB carcinoma was usually found heterogeneously enhanced in the arterial phase and commonly showed tortuous vascular distribution [26, 30]. When we focused on the blood flow and enhancement pattern on GB lesions, our result demonstrated that inhomogeneous enhancement on CEUS was not a promising indicator of malignancy with a relatively low sensitivity of 0.69, whereas the sensitivity through CH-EUS was 0.94. These findings suggest that enhancement imaging alone on CEUS seems to have only a limited value in the differential diagnosis of GB carcinoma and benign diseases, and given the possibility of the missed diagnosis, it is suggested that this pattern classification of CEUS should be an adjunct to final decision. Nevertheless, the observed enhancement pattern on the screen was a subjective judgment based on visual assessments. It’s supposed that the interpreters’ experience and different imaging resolution might cause heterogeneity. To some extent, a lesion could be presented more clearly through CH-EUS from a closer position, which benefits the diagnosis accuracy based on enhancement patterns and is a likely explanation for the excellent sensitivity in the present study. Thus, considering the variability of observers and imaging resolution, whether enhancement pattern in the arterial phase could be helpful to the diagnosis performance of CEUS needed to be further investigated with a larger multiple sample size.

According to previous reports, malignant lesions usually grow complicated tralesional vascularity [25, 34]. Taking advantage of microvascular depiction on CEUS, we summarized the diagnostic values of individual studies based on vessel shape. The pooled sensitivity and specificity confirmed that irregular vessel shape was one of important indicators of malignancy (0.81 and 0.88, respectively), which was in agreement with previous studies. GB carcinoma was more likely to exhibit tortuous or branch-like vessels after enhancement, by contrast, benign lesions were often stratified with dotted or linear vessels. Several authors have proposed that the findings of branched type tumor vessels and destruction of GB wall on CEUS were indicative of cancer, and the sensitivity, specificity, and accuracy of CEUS were 75–100%, 76.9–100%, and 84.5–91%, respectively [2, 21, 26, 40]. Therefore, combining the previous and present results, CEUS allowed differentiation of GB malignancy from benign lesions according to the presence of vascularity.

The application of contrast time parameter is another approach for image interpretation, and the time value has been widely used for diagnosis of lesions in the liver and other organs [41, 42]. In this meta-analysis, the parameters of arrival time, time to peak, and washout time were evaluated on CEUS for the diagnosis of GB diseases. In terms of arrival time and time to peak, no significant differences were found on either malignant or benign lesions. However, GB carcinoma appeared having a higher tendency to get enhanced and to reach hyper-enhancement in a shorter time, when compared with benign GB diseases. The washout time, on the other hand, was significantly shorter in malignancy group (*P* = 0.003) and was determined to be valuable for the malignancy detection with a pooled sensitivity of 0.81. A “fast-in and fast-out” enhancement feature has been shown in the malignant lesions due to abundant intralesional blood supply [2, 30]. It’s supported here that, contrast agent washes out earlier may reveal a high possibility of malignancy, but there is an absence of evidence to elucidate that earlier arrival of contrast agent can be a malignant feature of a lesion. On the other hand, the cut off value 28 s was directly determined by the smallest value among the included studies. This threshold of washout time deserves further evaluation, and the final diagnostic value may be higher.

To develop clinical practice, there are some earlier studies systematically assessing the accuracy of CEUS or other methods in detection of GB carcinomas by meta-analysis. (Table 3) Wang et al. included 16 studies and drew a similar conclusion that CEUS is a reliable imaging modality with a high sensitivity (0.91) and specificity (0.92) [43]. We found the pooled sensitivity of Wang et al. was higher than ours (0.92 vs. 0.81), and a possible explanation might be that the included studies in the two meta-analysis were different because Wang et al. also analyzed those studies in Chinese which we excluded because of larger publication bias. Cheng et al. also stated the same conclusion after data synthesis of 12 studies and generated a sensitivity of 0.81 and a specificity of 0.87 which were almost same as ours [44]. On the other hand, Myung-Won and Seong Jong focused on Diffusion Weighted Imaging and were the first to make a systematic reviews by combining 8 papers, and they found that Diffusion Weighted Imaging can discriminate malignant from benign GB lesions with excellent diagnostic performance in both qualitative and quantitative assessments [45]. Moreover, the current study was the first study to assess CH-EUS by meta-analysis. Obviously, evidence in this field is still limited and more relevant studies are required.

**Table 3:** Comparisons Among the Meta-analysis Assessing Different Methods for Differentiating Benign and Malignant Gallbladder Lesions

Authors	Proposed methods	Included studies	Evaluation measures	Statistical analyses	Results	Advantages	Disadvantages
Myung-Won and Seong Jong	Diffusion Weighted Imaging	8	Sensitivity, specificity, HSROC curve	Stata 10.0, R software 3.4.1	Sensitivity: 0.91 (95% CI: 0.91–0.91); specificity: 0.87 (95% CI: 0.87–0.87); HSROC curve: 0.95 (95% CI: 0.93–0.97).	Non-invasive, objective	Inefficient
Wang, et al.	CEUS	16	Sensitivity, specificity, PLR, NLR, DOR, HSROC curve	Stata 11.0, Review Manager 5.0	Sensitivity: 0.92 (95%CI: 0.90, 0.94); specificity: 0.91 (95%CI: 0.89, 0.93); PLR: 10.01 (95%CI: 7.02, 14.29); NLR: 0.10 (95%CI: 0.07, 0.14); DOR: 123.02 (95%CI: 78.40, 193.03); HSROC curve: 0.9689 (95%CI: 0.9376, 0.9879).	Cost, non-invasive, no-radiation-exposure	Subject
Cheng, et al.	CEUS	12	Sensitivity, specificity, PLR, NLR, DOR, SROC curve	Stata 12.0	Sensitivity: 0.81 (95%CI: 0.77, 0.84); specificity: 0.87 (95%CI: 0.85, 0.89); PLR: 10.43 (95%CI: 4.57, 23.83); NLR: 0.19 (95%CI: 0.11, 0.33); DOR: 58.84 (95%CI: 32.39, 106.88); SROC curve: 0.9371.		
Liang, et al. (the present study)	CEUS; CH-EUS	21	Sensitivity, specificity, DOR, SROC curve	Stata 15.0	(CEUS) Sensitivity: 0.81 (95% CI: 0.75–0.86); specificity: 0.92 (95% CI: 0.86–0.95); DOR: 64 (95%CI: 32, 127); SROC curve: 0.90 (95% CI: 0.87–0.92). (CH-EUS) Sensitivity: 0.92 (95% CI: 0.86–0.95); specificity: 0.89 (95% CI: 0.69–0.97); DOR: 89 (95%CI: 22, 354); SROC curve: 0.92 (95% CI: 0.90–0.94).	(CEUS) Cost, non-invasive, no-radiation-exposure (CH-EUS) Cost, no-radiation-exposure, high-resolution	(CEUS) Subject (CH-EUS) Subject, invasive, inconvenient

*CEUS* contrast-enhanced ultrasound; *CH-EUS* contrast-enhanced harmonic endoscopic ultrasound; *CI* confidence interval; *HSROC* hierarchical summary receiver operating characteristic; *PLR* positive likelihood ratio; *NLR* negative likelihood ratio; *DOR* diagnostic odds ratio; *SROC* summary receiver operating characteristic

The number of studies focusing on CH-EUS is too small to preclude us from investigating more imaging features on CH-EUS. Compared with CH-EUS, CEUS attracts more attention possibly because it is used more commonly in clinical settings. Many patients may refuse CH-EUS due to its invasiveness and inconvenience. However, CH-EUS can provide high-resolution images and sometimes is recommended to some patients, such as fat people. In the present study, both CEUS and CH-EUS are established to be a promising technique for distinguishing benign from malignant GB diseases, but their diagnostic accuracy greatly depend on the experience of readers. Experienced readers always can make a more positive diagnosis than those inexperienced, and therefore final diagnosis should be determined by an interpreter with rich experience in this field. Furthermore, standard diagnostic criteria should be established as guidelines based on imaging features to improve clinical practice.

There are some limitations existing in our study. High heterogeneity among the selected studies was a major problem, especially in the CH-EUS group. Although meta-regression and subgroup analysis revealed the influence of some factors on overall results, there were still other variances, like patients basic characteristics, operator’s experience, and different machines. Meanwhile, the number of included studies in CH-EUS group was limited, which was not of interest in subgroup analysis and further investigation. Furthermore, all the analyzed studies were conducted in Asian area, which means geography could be a factor causing some bias in the final analysis. Because GB carcinoma is more common in Latin America and Asia, whereas it has significant low incident rate in the west countries [46]. Thus, future trails covering various countries with a larger sample size are encouraged to verify our results.

## Conclusions

The results of the present meta-analysis suggest that both CEUS and CH-EUS are promising and reliable imaging modalities for the differential diagnosis between malignant and benign GB lesions, with high sensitivity and specificity. Moreover, CH-EUS might be more sensitive for malignancy detection than CEUS. For CEUS, irregular tralesional vessels and washout time within 28 s are indicative of malignancy; either heterogeneous enhancement or discontinuity of GB wall are still not determined as diagnostic criteria for malignant lesions. For CH-EUS, heterogeneous enhancement is suggestive of GB malignancy. However, considering CEUS and CH-EUS are novel techniques in the GB diagnostic system, and concerning about the existing heterogeneity and limitations, their application should be cautious. In addition, more rigorous evidence in further studies is needed, especially about the comparison between CEUS and CH-EUS.

## Data Availability

The datasets used and/or analyzed during the current study are available from the corresponding author on reasonable request.

## Abbreviations

US: Ultrasound
CEUS: Contrast-enhanced ultrasound
CH-EUS: Contrast-enhanced harmonic endoscopic ultrasonography
GB: Gallbladder
MI: Mechanical index
TP: True-positive
TN: True-negative
FP: False-positive
FN: False-negative
DOR: Diagnostic odds ratio
AUC: Area under the curve
SROC: Summary receiver operating characteristics
WMD: Weighted mean differences
CI: Confidence intervals
QUADAS-2: The Quality Assessment of Diagnostic Accuracy Studies
